RETRACTED

# Oral health-related quality of life in rheumatoid arthritis: a comparative analysis

**DOI:** 10.1186/s41927-022-00292-w

**Published:** 2022-10-18

**Authors:** Amirhossein Parsaei, Aida Mehdipour, Hamidreza Ghadimi, Ashkan Mohammadi Kooshki, Parisa Shajari, Maryam Masoumi, Pouya Torabi, Hossein Azizi, Behnam Amini, Hanie Karimi, Hojat Dehghanbanadaki, Mohammad Aghaali, Soroush Moradi

**Affiliations:** 1 Faculty of Medicine, Tehran University of Medical Sciences, Tehran, Iran; 2 Qom Dental School, Qom University of Medical Sciences, Qom, Iran; 3 School of Medicine, Qom University of Medical Sciences, Qom, Iran; 4 School of Medicine, Iran University of Medical Science, Tehran, Iran; 5 Student Research Committee, School of Dentistry, Qom University of Medical Sciences, Qom, Iran; 6 Clinical Research of Development Center, Shahid Beheshti Hospital, Qom University of Medical Sciences, Qom, Qom Iran; 7 Endocrinology and Metabolism Research Center, Endocrinology and Metabolism Clinical Sciences Institute, Tehran University of Medical Sciences, Tehran, Iran; 8 Department of Community Medicine, School of Medicine, Qom University of Medical Sciences, Qom, Iran

**Keywords:** Rheumatoid arthritis, OHIP-14, OHRQol, Oral health, DAS28, Rheumatology

## Abstract

**Background:**

Compared to the healthy population, the psychological impact of rheumatoid arthritis(RA) on patients' lives could dramatically lower their oral health-related quality of life (OHRQoL). Our goal is to analyze OHRQoL in RA patients and look into the role of disease activity, dental health index, and Temporomandibular disorders score in maintaining their oral health.

**Methods:**

In a cross-sectional comparative study, we compared a sample of 40 RA patients with 40 age- and gender-matched healthy controls in terms of oral health and OHRQoL. Temporomandibular disorders (TMD), number of decayed, filled, or missing teeth (DMFT), and Oral Health Impact Profile (OHIP) were among the oral health factors studied (OHIP-14). This study also looked at the link between the RA disease activity score (DAS28) and oral health factors.

**Results:**

RA patients had a significantly higher mean (poorer OHRQol) than healthy controls in total oral function, total psychosocial impact, OHIP-14 sum score, OHIP-14 extent score, TMD score and the number of missed teeth (Mann–Whitney U test, *P*-value < 0.05). After adjustment for DMFT, only the oral function score of OHIP-14 had a significant correlation with disease activity (Mann–Whitney U test, *P*-value < 0.05). The TMD sum score significantly correlated with disease activity regardless of adjustment for DMFT (Spearman's Correlation test, *P*-value < 0.05 for both). The number of decayed teeth and missed teeth showed a positive correlation with increased disease activity (Coefficient = 0.239 and 0.245, *P*-value < 0.05 for both).

RETRACTED

**Conclusions:**

Patients with RA are less satisfied with their oral health than healthy controls. In RA patients, the number of missing teeth and temporomandibular disorders was substantially greater, and the number of missing teeth and temporomandibular diseases increased significantly with increased disease activity. Although OHRQoL was inversely connected with RA activity, after correcting for decaying, missing, and filled teeth, only the oral function score of OHIP-14 exhibited a slight connection to DAS28.

**Supplementary Information:**

The online version contains supplementary material available at 10.1186/s41927-022-00292-w.

## Introduction

Rheumatoid Arthritis (RA) is a chronic autoimmune condition manifesting with the inflammation of joints and synovial surfaces [1]. With approximately 1% of the worldwide population affected by this autoimmune disease, RA can lead to joint destruction, severe movement limitations, and death if it remains untreated [2]. Early diagnosis of RA and proper treatment could decrease its complications and enhance patients' ability to perform daily tasks [3]. The treatment regimen for RA usually consists of corticosteroids and disease-modifying antirheumatic drugs (DMARDs) [4].

Health-related quality of life (HRQoL) seems to be decreased in RA patients [5]. Pain and movement limitations caused by the universal inflammatory process, disease burden, and psychosocial impact on patients' lives could significantly reduce their HRQoL compared to the healthy population [6]. RA's inflammatory activities in the orofacial region involve the temporomandibular joint (TMJ), which plays an essential role in food consumption and verbal abilities [7]. Temporomandibular disorder (TMD) could restrict patients' capacity in eating and speaking [8]. Furthermore, previous studies demonstrated a correlation between RA and the inflammation of gingiva and periodontium [9]. Both periodontitis and RA begin with inflammation of the soft tissues and progress to bone structural damage and loss of function [10]. The local microbiome is altered in periodontitis, increasing periodontopathic bacteria such as Porphyromonas gingivalis [10, 11]. Bacterial growth and periodontitis were higher in persons at risk of RA before joint symptoms [11].

Oral Health-related quality of life (OHRQoL), as one of the major sub aspects of HRQoL, has been discussed recently in the literature [7, 12, 13]. Although previous studies demonstrated orofacial involvement in RA patients, the impact of these complications on OHRQoL remains ambiguous. Our study aims to assess Oral Health-Related Quality of Life (OHRQoL) via OHIP-14 questionnaire in RA patients and investigate the possible impact of different clinical parameters, including disease activity, number of decayed, filled, or missing teeth (DMFT), and TMD, in their oral health maintenance.

RETRACTED

## Methods

### Study design and participants

This research is a cross-sectional, comparative study conducted between September 2021 and January 2022 at a large urban hospital center (Shahid Beheshti hospital), Qom, Iran. The study protocols were designed according to the Strengthening the Reporting of Observational Studies in Epidemiology (STROBE) statement.

We recruited a consecutive sample of RA patients diagnosed with RA from the Shahid Beheshti hospital rheumatology clinic during the study period by expert attends of the rheumatology department. The inclusion criteria were age > 18 years and consent for participation. We excluded RA patients with other rheumatologic, systemic or autoimmune diseases, active infection, inflammatory conditions, endocrine disorders or malignancies and pre-existing oral disorders unrelated to RA (Oral herpes, oral malignancies, bacterial and fungal infections and other diagnosed inflammatory disorders). The patients who had one of the mentioned conditions were excluded according to the consultation and evaluation by the second specialist. The control group was selected from a consecutive sample of parents who visited the vaccination clinic of the same hospital to give their children routine vaccination shots. The controls were matched for gender and age ± two years.

The participants were examined and interviewed by one expert rheumatologist and one expert dentist for demographic (age, gender, education, employment status, marital status), medical history, and clinical data. The medical and clinical data included disease duration and severity, oral and dental examination, temporomandibular disease examination, oral health-related quality of life assessment, medication history and laboratory data. Informed consent was taken from all participants.

### Diagnosing and severity assessment of RA

The patients were diagnosed with RA according to ACR/EULAR 2010 criteria for rheumatoid arthritis classification be an expert rheumatologist [14]. We used DAS28 [15] score to label RA activity in patients to remission (DAS28 < 2.6), low (2.6 ≤ DAS28 < 3.2), moderate (3.2 ≤ DAS28 ≤ 5.1) and high (5.1 < DAS28). DAS28 score was calculated using the "das-score" online calculator [16] based on four measures, including the number of tender joints, the number of swollen joints, the blood level of ESR(mm/hr) and visual analog scale (VAS) of patient's general health (mm).

RETRACTED

### Oral health-related quality of life assessment

We used Oral Health Impact Profile (OHIP-14) during interviews to assess the participants' oral health-related quality of life. The validated version of OHIP-14 consists of 14 items in seven dimensions: functional limitation, physical discomfort, psychological discomfort, physical disability, psychological disability, social disability, and handicap [17]. The score for each item is recorded in the form of a Likert scale: 0(never), 1(hardly ever), 2(occasionally), 3(fairly often) and 4(very often). The OHIP-14 sum score is the sum of all items ranging from 0 to 56; The OHIP-14 extent score is the total number of questions that had scores 3 or 4(fairly often and very often) ranging from 0 to 12 [18]. Higher scores of OHIP-14 represent a higher overall burden of oral health-related quality of life. Based on Schmalz et al. [19] the total oral function is a dimension that is the sum of items”trouble pronouncing words”, “Sense of taste worsened”, “interrupt meals”, “uncomfortable eating” and “diet unsatisfactory”. Total psychosocial impact is the sum score of items “life less satisfying”, “difficulty relaxing”, “felt tense”, “irritable with other people”, “difficulty doing usual jobs”, “unable to function” and “being embarrassed”.

### Oral health examination and temporomandibular joint disorders

One expert dentist and one rheumatologist examined and interviewed patients for dental health and temporomandibular disorders (TMD). The dental examination consisted of the number of decayed, missing and filled teeth represented as DMFT (sum of all three measures). The TMD was measured using a researcher-designed questionnaire with 13 items that demonstrate the patient's extent of discomfort (Additional file 1: Table 1). The questions are subject to different aspects of TMD, including clicks, discomfort, pain, limitation in movement, chewing, and swallowing. The questions are in the form of a Likert scale with scores of 0(never), 1(sometimes), 2(often) and 3(always). The total TMD score ranges from 0 to 52, and a higher score represents a higher extent of TMD.

### Bias

The risk of bias for the clinical judgment was limited by the clinician's judgment according to ACR/EULAR system. The assessment of dental findings using DMFT, OHRQoL using OHIP-14 in the form of a likert scale, and TMD using formal questionnaires and reporting the results in numbers reduced the possibility of misinterpretation. Laboratory tests were also analyzed in an exclusive laboratory in Shahid Beheshti hospital. If participants had inconsistent clinical and paraclinical assessments, the participant was re-assessed for a second time, and the latter was reported.

RETRACTED

### Statistical analysis

Continuous variables were presented as mean ± standard deviation (SD), and categorical variables were described in frequency and percentage in the form of tables. Categorical variables were compared between groups using Fischer's Exact test. Preliminary analyses showed no outliers, as assessed by boxplot. The continuous variables were tested for normality using the Shapiro–Wilk's test; data that did not meet assumptions for parametric tests, including variables without normal distribution (Shapiro–Wilk's test (*P* < 0.05)) were compared between two independent groups with Mann–Whitney U test and between more than two groups with Kruskal–Wallis test.; the Man-Whitney U test assumption of equal distribution were tested by using Levene's test for equality of variances based on median and with an adjusted degree of freedom. To detect correlations between clinical and medical variables and disease activity (DAS-28 score) in RA patients, Spearman's rank correlation coefficient was applied with and without adjustment for DMFT. According to Cohen 1988, the effect size of correlations was interpreted as small (0.1–0.3), medium (0.3–0.5) or large (> 0.5) [20]. Statistical analysis was performed using SPSS, Version 26.0 (SPSS Inc., USA.).

## Results

### Participants' characteristics

Table 1 compared forty RA patients and forty age/gender-matched healthy controls for demographic and medical characteristics. The patients and controls are comparable regarding marital status, education, job and smoking (Fischer's Exact test, *P*-value > 0.05). The RA patient's most used medications were prednisolone (97.5%) with mean dose of 5.5, methotrexate (77.5%) and hydroxychloroquine (55%) and the disease duration was 5.7 ± 6.3 years.

**Table 1:** Demographic and medical characteristics of Participants

	Controls N = 40	RA patients N = 40	*P*-value*
Age (years), Mean ± SD	53.3 ± 8.2	53.7 ± 7.8	0.824
*Gender, N(%)*			
Female	34 (85)	34 (85)	–
Male	6 (15)	6 (15)	
*Marital status, N(%)*			
Not married	1 (2.5)	2 (5)	1.000
Married	39 (97.5)	38 (95)	
*Education, N(%)*			
Middle school or lower	32 (80)	27 (67.5)	0.151
Secondary school	3 (7.5)	8 (20)	
Diploma	3 (7.5)	1 (2.5)	
Bachelor's degree	1 (2.5)	4 (10)	
Master's degree	0	0	
Doctorate or higher	1 (2.5)	0	
*Job, N(%)*			
Housewife/unemployed	30 (75)	30 (75)	0.514
Full-time employee	4 (10)	1 (2.5)	
Self-employed	4 (10)	5 (12.5)	
Retired	2 (5)	4 (10)	
*RA medications, N(%)*			
Prednisolone		39 (97.5)	–
Methotrexate		31 (77.5)	
Hydroxychloroquine		22 (55)	
Leflunomide		9 (22.5)	
Sulfasalazine		3 (7.5)	
Adalimumab		3 (7.5)	
Methylprednisolone acetate		2 (5)	
Etanercept		2 (5)	
Prednisolone dose (mg/day), Mean ± SD		5.7 ± 2.2	–
Positive Anti-citrullinated protein antibody, N(%)		13 (65)	–
Smoking, N(%)	4 (10)	6 (15)	0.749
Disease duration (years), Mean ± SD		5.7 ± 6.3	–
Positive rheumatoid factor, N(%)		4 (10)	–
Remission (DAS28 < 2.6)		15 (37.5)	–
*Disease activity, N(%)*			
Low (2.6 ≤ DAS28 < 3.2)		7 (17.5)	
Moderate (3.2 ≤ DAS28 ≤ 5.1)		12 (30)	
High(5.1 < DAS28)		6 (15)	

*Fischer's exact or independent samples t-test as appropriate

RETRACTED

### Oral health-related quality of life in RA patients vs. healthy controls

As Table 2 demonstrates, RA patients scored significantly higher mean scores (lower quality of life) than healthy controls in total oral function, total psychosocial impact, OHIP-14 sum score and OHIP-14 extent score (Mann–Whitney U test, *P*-value < 0.05). The mean scores of each OHIP-14 item are compared between RA patients and healthy controls in detail. RA patients had higher mean scores than healthy controls regarding items "Trouble pronouncing words", "Sense of taste worsened", "Uncomfortable eating", "Felt self-conscious", "Felt tense", "Diet unsatisfactory", "Difficulty relaxing", "Been embarrassed", "Difficulty doing usual jobs", "Life less satisfying" and "Unable to function" (Mann–Whitney U test, *P*-value < 0.05 for all items).

**Table2:** Comparison of Oral Health Impact Profile scores between RA patients and healthy controls(left), and assessment of the association of each item with RA activity(right)

OHIP-14 dimensions/questions	Mann–Whitney U test					Kruskal–Wallis test				
	Study groups, mean ± SD					RA activity, mean rank				Significance
	Control(N = 40)	RA patients(N = 40)	Total(80 N)	Z-score	Significance	Remission	Low Disease Activity	Moderate Disease Activity	Severe Disease Activity	
Trouble pronouncing words	0.08 ± 0.35	0.42 ± 0.93	0.25(0.72	−2.275	.023*	19.93	16.00	24.63	18.92	0.170
Sense of taste worsened	0.43 ± 0.74	1.25 ± 1.37	0.84 ± 1.17	−2.954	.003*	19.97	19.00	21.67	21.25	0.956
Painful aching in mouth	0.90 ± 0.92	1.33 ± 1.24	1.11 ± 1.11	−1.415	0.157	19.87	16.29	24.13	19.75	0.507
Uncomfortable eating	0.35 ± 0.77	1.33 ± 1.45	0.84 ± 1.25	−3.331	0.001*	23.33	17.36	22.63	12.83	0.171
Felt self-conscious	0.50(0.96	1.15 ± 1.36	0.83 ± 1.22	−2.367	0.018*	22.83	18.64	22.08	13.67	0.314
Felt tense	0.30 ± 0.79	1.00 ± 1.39	0.65 ± 1.18	−2.750	0.006*	21.97	20.71	21.63	14.33	0.474
Diet unsatisfactory	0.20 ± 0.56	0.78 ± 1.25	0.49 ± 1.00	−2.313	0.021*	21.33	22.57	19.96	17.08	0.750
Interrupt meals	0.37 ± 0.62	0.70 ± 1.06	0.54 ± 0.88	−1.300	0.194	20.53	21.29	21.42	17.67	0.901
Difficulty relaxing	0.27 ± 0.64	1.00 ± 1.377	0.64 ± 1.12	−2.776	0.006*	22.70	23.93	20.25	11.50	0.128
Been embarrassed	0.30 ± 0.68	1.08 ± 1.52	0.69 ± 1.23	−2.336	0.019*	19.83	23.00	23.88	12.50	0.147
Irritable with other people	0.38 ± 0.58	0.80 ± 1.32	0.59 ± 1.04	−.674	0.501	21.23	19.79	20.46	19.58	0.981
Difficulty doing usual jobs	0.18 ± 0.44	0.63 ± 1.17	0.40 ± 0.90	−1.623	0.105	22.37	21.00	19.29	17.67	0.701
Life less satisfying	0.10 ± 0.37	0.75 ± 1.29	0.43 ± 1.00	−2.874	0.004*	21.13	20.29	23.08	14.00	0.307
Unable to function	0.15 ± 0.36	0.58 ± 1.15	0.36 ± 0.87	−1.393	0.164	21.30	21.43	20.08	18.25	0.894
Total Oral Function	1.42 ± 2.17	4.47 ± 4.49	2.95 ± 3.82	−3.592	< 0.001*	20.93	19.86	22.42	16.33	0.766
Total Psychosocial Impact	1.67 ± 2.30	5.82 ± 8.06	3.75 ± 6.25	−1.709	0.087	20.20	23.00	23.25	20.20	0.286
OHIP-14 sum score	4.50 ± 5.49	12.78 ± 14.04	8.64 ± 11.38	−3.186	0.001*	20.60	19.57	23.21	15.92	0.655
OHIP-14 Extent score	0.30 ± 0.88	1.98 ± 3.48	1.14 ± 2.66	−2.874	0.004*	20.97	23.07	21.21	14.92	0.518

*Statistically significant difference (*P*-value < 0.05)

The mean score of OHIP-14 items showed no association with DAS-28 categories in RA patients (Kruskal–Wallis test, *P*-value > 0.05 for all items).

RETRACTED

### Oral and dental characteristics in RA patients vs. healthy controls

As Table 3 shows, RA patients had significantly higher TMD sum scores than healthy controls (Mann–Whitney U test, *P*-value < 0.001). The mean number of Missed teeth in RA patients is 9.60 ± 8.98, which is significantly higher than 5.07 ± 5.53 in healthy controls (Mann–Whitney U test, *P*-value = 0.16). The TMD score, number of decayed, missed or filled teeth showed no association with DAS-28 categories (Kruskal–Wallis test, *P*-value > 0.05 for all items).

**Table 3:** Comparison of temporomandibular joint disorder and DMFT between RA patients and healthy controls(left), and assessment of the association of each item with RA activity(right)

Items	Mann–Whitney U					Kruskal–Wallis				
	Study groups					RA activity				
	Control(40 N)	RA patients(40 N)	Total(80 N)	Z-score	Significance	Remission	Low Disease Activity	Moderate Disease Activity	Severe Disease Activity	Significance
TMD sum score	2.05 ± 1.89	6.67 ± 7.59	4.36 ± 5.97	−4.433	< 0.001	19.03	19.21	24.71	17.25	.500
Decayed Teeth	2.00 ± 1.93	3.95 ± 3.95	2.97 ± 3.24	−1.852	.064	19.13	18.79	22.58	21.75	.842
Missed Teeth	5.07 ± 5.53	9.60 ± 8.98	7.34 ± 7.34	−2.420	.016*	22.30	18.43	17.88	23.67	.652
Filled Teeth	3.45 ± 3.85	3.80 ± 4.83	3.63 ± 4.34	−.304	.761	21.97	17.71	21.33	18.42	.817

*Statistically significant difference (*P*-value < 0.05)

### Correlation between disease activity and clinical and medical variables

The oral function score of OHIP-14, OHIP-14 sum score and OHIP-14 extent score showed a significant correlation with higher disease activity (Spearman's coefficient = 0.373, 0.330 and 0.263 respectively, *P*-value < 0.05 for all). However, after adjustment for DMFT, only the oral function score of OHIP-14 had a significant correlation with disease activity(*P*-value < 0.05).

RETRACTED

The TMD sum score significantly correlated with disease activity regardless of adjustment for DMFT (Spearman's Correlation test, *P*-value < 0.05 for both).

Between three items of DMFT, the number of decayed teeth and number of missed teeth showed a positive correlation with increased disease activity (Coefficient = 0.239 and 0.245, *P*-value < 0.05 for both) (Table 4).

**Table 4:** Correlation between clinical and medical variables and disease activity in RA patients, with and without adjustment for DMFT

Variables	Spearman’s correlation	
	No adjustment	After adjustment for DMFT
	DAS-28 score	DAS-28 score
*Oral function*		
Coefficient	0.373*	0.241*
Significance	0.001	0.033
*Psychosocial impact*		
Coefficient	0.160	0.091
Significance	0.158	0.429
*OHIP-14 sum score*		
Coefficient	0.330*	0.149
Significance	0.003	10.192
*OHIP-14 extent score*		
Coefficient	0.263*	0.103
Significance	0.018	0.370
*TMD sum score*		
Coefficient	0.477*	0.246*
Significance	< 0.001	0.030
*Decayed teeth*		
Coefficient	0.239*	–
Significance	0.033	–
*Missed teeth*		
Coefficient	0.245*	–
Significance	0.028	–
*Filled teeth*		
Coefficient	−0.056	–
Significance	0.622	–

*Significant correlation by Spearman's test, *P*-value < 0.05

## Discussion

Rheumatoid Arthritis, as a chronic systemic disorder, decreases the overall health-related quality of life compared to the general population and mainly due to their physical limitations and pain [21]. Although previous studies have agreed upon this conclusion [6, 12, 18, 22], the literature remains controversial in assessing specific aspects of HRQoL. As one of these aspects, dental health and oral hygiene in RA patients have been discussed in numerous studies [12, 13, 23–26]. Our study aims to assess Oral Health-Related Quality of Life (OHRQoL) via OHIP-14 questionnaire in RA patients and investigate the possible impact of different clinical parameters, including disease activity, DMFT index, and TMD score, in their oral health maintenance.

Our results revealed that RA patients were significantly less convenient with their oral health than healthy controls. These patients had more negative perceptions about their total oral function and its psychosocial impact. However, we found no significant correlation between disease activity (based on the DAS28 score) and OHRQoL (mean score of OHIP-14 items) in RA patients. They had more negative preception about their temporomandibular function (TMD sum score) and significantly more missed teeth than the control group. The oral function score of OHIP-14, OHIP-14 sum score, and OHIP-14 extent score significantly correlated with disease activity.

RETRACTED

Moreover, the number of decayed and missed teeth (based on the DMFT index) positively correlated with RA activity. Since the number of missing or decayed teeth greatly impacts individuals ' perception of oral health, we adjusted our desired variables based on the DMFT score. After the adjustment, only the oral function score of OHIP-14 and TMD score remained significantly correlated to RA activity.

RA patients seem to be more concerned about their oral health quality. As previous studies suggest, physical limitations and pain caused by the disease restrict patients' ability to maintain their dental hygiene. In a large study in Finland 2014, 564 RA patients and 431 controls were compared based on their response to the OHIP-14 questionnaire [24]. Ahola et al. found that the mean total score was significantly higher in RA patients, which means they're less satisfied with their oral health condition. In 2017, Mühlberg et al. compared OHRQoL (with a german short version of OHIP-14) between 103 RA patients and 104 age and gender-matched healthy controls [26]. Although they found significantly worse OHRQoL in RA patients, their clinical assessment and dental examination revealed no considerable difference in DMFT or periodontitis prevalence. Schmalz et al.'s survey on 176 RA patients in 2020 found no significant difference in their OHIP-14 scores compared to reference values for the healthy population [19]. However, the psychosocial dimension (*P*  = 0.017) the OHIP-14 sum scores (*P* = 0.041) showed a positive correlation with DAS28-ESR. In the present study, RA patients reported significantly higher scores for OHIP-14 rather than healthy controls. While our patients were not happy with their OHRQoL, the mean score of OHIP-14 items showed no association with DAS-28. These results could indicate that RA patients have more negative perceptions about their OHRQoL than the control group, regardless of disease activity score.

Previous studies reported Temporomandibular involvement and diseases of TMJ are more prevalent in RA patients. Since this mobile joint largely impacts persons' ability to eat and speak, the TMJ range of motion impairment could negatively affect their perceptions about oral health. Cristina et al. in 2018 assessed TMJ involvement in 135 RA patients and investigated its correlation with disease activity (DAS28-ESR) and quality of life [25]. TMJ involvement was observed in one-third (29.61%) of their patients and positively correlated with disease activity and reduced quality of life. Ahmed et al. also found the same result in a study on 33 RA patients with TMJ involvement in 2013 [23]. The present study results indicate RA patients with significantly higher TMD scores than controls are not satisfied with their temporomandibular function. In line with previous studies, further analysis revealed a positive correlation of TMD sum scores with disease activity. Besides TMD, tooth loss also plays a major role in oral health. Previous studies on healthy participants reported that a large number of missing teeth significantly reduces OHRQoL. Schmalz et al. found that RA patients are likely to have more missing teeth than controls, and it is directly associated with increased OHIP-G14 scores and, therefore, poorer OHRQoL [19]. In the present study, the number of missing teeth was also significantly higher in RA patients, resulting in higher OHIP-14 scores, and it was positively correlated with disease activity. However, our result contrasts with Mühlberg et al.'s study. They found no significant difference in DMF-T index between RA and control group and no specific correlation of missing teeth to OHRQoL in RA patients [26].

RETRACTED

RA activity seems to decrease patients' quality of life. The literature suggests that patients with a more progressive RA experience further limitations and pain in daily life routine. Radwan-Oczko et al., in a study in 2020, investigated OHRQoL in 164 patients with RA [22]. They found that a higher level of DAS28 was significantly associated with pain or discomfort in the oral cavity, which negatively impacts patients' perceptions of their oral health, especially in younger ages. Schmalz et al. also found this significant correlation between DAS28-ESR and OHIP-G14 sum scores [19]. However, Monsarrat et al. in the OSARA study were unable to find any significant correlation between disease activity and dental health in RA patients [27]. Mühlberg et al. also found no considerable correlation between DAS28 and RA patients' dental findings [26]. Our initial analysis revealed the oral function score of OHIP-14, OHIP-14 sum score, and OHIP-14 extent score significantly correlated with disease activity. Since the number and missing or decayed teeth greatly influence an individual's oral health and following controversial findings in the literature, we decided to adjust our desired variables based on the DMFT index. After the adjustment for DMFT, only the oral function score of OHIP-14 weakly (*P* = 0.033) correlated with disease activity. This result could indicate that patients with higher disease activity are less satisfied with their oral function, regardless of their dental findings. Previous studies suggested that RA patients with higher disease activity have difficulties maintaining dental hygiene, especially toothbrushing [28].

RETRACTED

We recommend future prospective studies to assess oral health in a larger sample size from multiple centers. We also suggest the use of other dental indices and examinations be investigated in OHRQoL of RA patients. Since socioeconomic status and psychological traits play a major role in conserving dental health, we strongly suggest investigating these parameters in RA patients. In the current study Although we tried to exclude RA patients with pre-existing oral disorders, but distinction of oral findings that are related to RA from those that are unrelated to RA is not definite. In the current study the TMD examinations was performed by rheumatologists. It would have been interesting to investigate whether the TMD discomfort reported by patients with RA could be justified or explained by an objective TMD disfunction assessed on physical examination by a dedicated specialist (e.g., masticatory muscles palpation, deviations, clicks during mandibular movements). We suggest future studies to take this point into consideration to achieve a more acurate assessment of TMD discomfort. It is worth noting that the authors of this work did not explore TMD in the study population (i.e. prior or current temporo-mandibular joint arthritis), which may result in an inescapable bias in the assessment of Temporomandibular related discomfort in the patients. Our participants received a variety of medications that could affect their oral health. We also recommend future studies to assess how RA patients' medications, especially immunosuppressors and immunomodulators, impact their OHRQoL. In light of the potential importance of periodontitis in RA patients' dental health-related quality of life, we recommend that future studies look into periodontitis in a similar sample of RA patients.

The current study confirms the previous finding of decreased OHRQoL in RA patients compared to healthy individuals. Furthermore, assessing TMD as a secondary component of Oral discomfort in RA patients in addition to DMFT and OHIP-14 creates a full spectrum of possible aspects of how this population is affected. In the history of research, the current type of studies (quality of life) has received less attention and funding in less developed countries, including Iran. Regarding the country's race and genetics, current results create a more balanced understanding of what literature provides about this subject. The importance of this article is that it paves the way for future studies to improve the quality of life in rheumatoid arthritis patients.

RETRACTED

## Conclusion

In conclusion, RA patients are less pleased with their oral health quality than healthy controls. The number of missing teeth and temporomandibular diseases were significantly higher in RA patients, and they were significantly increased with higher disease activity. Although OHRQoL negatively correlated with RA activity, only the oral function score of OHIP-14 had a weak correlation to DAS28 after adjusting for decayed, missed, and filled teeth.

## Supplementary Information

**Additional file 1. Table 1**. Temporomandibular joint disorder questionnaire.

## Data Availability

The data that support the findings of this study are available from Qom University of Medical Sciences but restrictions apply to the availability of these data, which were used under license for the current study, and so are not publicly available. Data are however available from the corresponding author (Maryam Masoumi) upon reasonable request and with permission of Qom University of Medical Sciences.

## Abbreviations

DAS: Disease activity score
DMARDs: Disease-modifying antirheumatic drugs
DMFT: Decayed, missing or filled teeth
HRQoL: Health-related quality of life
OHIP: Oral Health Impact
OHRQoL: Oral health-related quality of life
RA: Rheumatoid arthritis
STROBE: Strengthening the reporting of observational studies in epidemiology
TMD: Temporomandibular disorder
TMJ: Temporomandibular joint
